# Performance Comparison of GeneXpert MTB/RIF, Gene Chip Technology, and Modified Roche Culture Method in Detecting *Mycobacterium tuberculosis* and Drug Susceptibility in Sputum

**DOI:** 10.1155/2022/2995464

**Published:** 2022-07-18

**Authors:** Changli Xie, Xin Hu, Yali Liu, Chengfeng Shu

**Affiliations:** Medical Laboratory, Bishan District People's Hospital of Chongqing, Chongqing, China

## Abstract

Our aim of this study was to observe and analyze the performance of the real-time fluorescence quantitative nucleic acid amplification detection of *Mycobacterium tuberculosis*/rifampicin resistance (GeneXpert MTB/RIF), gene chip technology, and modified Roche culture method in detecting MTB in sputum submitted for inspection and drug susceptibility. Patients with smear-negative suspected pulmonary TB (*n* = 120) in our hospital were enrolled in this study using a random number table, and sputum samples submitted for inspection were tested by the GeneXpert MTB/RIF, gene chip technology, and modified Roche culture method. With clinical diagnosis as the gold standard, the performance (mainly sensitivity and specificity) of the above three detection methods in the diagnosis of MTB was compared. Next, the drug susceptibility test (DST) was carried out on sputum samples, tested positive by the three methods. With the solid culture results as the evaluation criteria, the performance of the three detection methods in the diagnosis MTB and DST was compared. When compared with the modified Roche culture method, the GeneXpert MTB/RIF had the highest positive rate and a shorter overall test duration (*P* < 0.05). In contrast with the gene chip technology, the GeneXpert MTB/RIF exhibited higher sensitivity and negative predictive value (NPV) and lower specificity, accuracy, positive predictive value (PPV), and Kappa value (*P* < 0.05). According to analysis of the diagnostic performance of the three detection methods, GeneXpert MTB/RIF displayed the highest diagnostic sensitivity, ideal predictive values, and the highest similarity with clinical diagnosis in results (*P* < 0.05). The detection of susceptibility to isoniazid (INH) and RIF showed that the GeneXpert MTB/RIF and gene chip technology performed ideally in DST of MTB. In comparison with the modified Roche culture method, the GeneXpert MTB/RIF and gene chip technology have more prominent performance in detecting MTB and drug susceptibility. Besides, to further improve the accuracy of clinical diagnosis, various molecular biology detection methods can be combined to avoid delaying of the best time for the diagnosis and treatment of the disease.

## 1. Introduction

Tuberculosis (TB) is one of the major social and public health problems all over the world. In China, one of the twenty-two countries with a high TB burden, multidrug-resistant TB emerges and spreads, bringing new challenges to the prevention and control of TB therein [1]. The drug susceptibility test (DST) used previously is usually performed on the basis of culture. In brief, strains are cultured and then isolated for a relatively long time (about 3–8 weeks), and on this basis, final DST results are obtained about one month later [2, 3]. As a result, the previous drug sensitivity test (DST) took a relatively long time to perform and was not effective in providing clinicians with timely and scientifically sound results for diagnosing patients' diseases. As molecular biology diagnostic technologies are adopted in clinical tests, more advanced detection methods are widely applied in the laboratory detection of TB, among which the real-time fluorescence quantitative nucleic acid amplification detection of MTB/RIF resistance (GeneXpert MTB/RIF) and gene chip technology are frequently used at this stage [4]. Through a search of the current published literature, the lesser literature compares the diagnostic efficacy of the GeneXpert MTB/RIF (real-time quantitative fluorescent nucleic acid amplification assay), the gene chip technique, and the modified Roche culture method for sputum sent for testing, respectively. Based on this, in this work, the GeneXpert MTB/RIF, gene chip technology, and modified Roche culture method were employed to detect the sputum submitted for inspection, respectively, and their performance in detecting TB and drug susceptibility was observed and analyzed.

## 2. Patients and Methods

### 2.1. Patients

A total of 120 patients with smear-negative suspected pulmonary TB in our hospital were enrolled in this study using a random number table, and sputum samples submitted for inspection were detected by the GeneXpert MTB/RIF, gene chip technology, and modified Roche culture method. The 120 patients were mainly aged 22–73 years, with a mean of (55.54 ± 17.75) years, and the ratio of males to females was 64/57. The basic data showed no statistically significant differences (*P* > 0.05), worthy of further comparative analysis. The inclusion criteria were set as follows: patients were included in this study based on their clinical treatment history, symptoms, and final results of a series of examinations (immunological detection, detection of sputum smear samples sent for inspection, and imaging examination). The final clinical diagnosis indexes of TB were assessed by observing and analyzing whether the culture or histopathological test results are positive or significant efficacy is obtained after administration of antituberculosis drugs. TB was diagnosed according to clinical guidelines [5]. The inclusion criteria were set as follows: patient was <18 years old, patient had a positive sputum smear, and patient had severe hepatic and renal insufficiency. According to the final diagnosis, the ratio of TB patients to non-TB patients was 78 : 42.

### 2.2. Methods

Three sputum samples (the first sputum) were collected in the early morning from each patient enrolled in this study in time, with a sample size of 5 mL for each sample. Then, clinical tests were carried out, after which two samples with a higher positive grade (higher than 2^+^) were selected. Next, 1 mL each of sputum was collected from the two samples, mixed well, and tested in time. The positive grade of smears was assessed based on the following criteria: no acid-fast bacilli observed after continuous observation of 300 different fields of view suggested negative, 1–8 acid-fast bacilli observed after continuous observation of 300 different fields of view indicated suspected positive, 3–9 acid-fast bacilli observed after continuous observation of 100 different fields of view suggested 1^+^, 1–9 acid-fast bacilli observed after continuous observation of 10 different fields of view indicated 2^+^, 1–9 acid-fast bacilli observed after continuous observation of 1 field of view indicated 3^+^, and 10 acid-fast bacilli observed in each field of view indicated 4^+^.

#### 2.2.1. Modified Roche Culture Method

Sputum samples treated were inoculated into an acidic modified Roche medium and timely placed in a constant temperature incubator for bacterial culture. At the 3 d after inoculation, the medium was observed for the presence of MTB, followed by observation once a week until the eighth week after inoculation. No MTB observed indicated a negative result. If MTB was observed, a combined report analysis was performed in combination with the actual growth status of MTB in the culture medium. MTB strains were subjected to DST in a proportional manner.

#### 2.2.2. GeneXpert MTB/RIF

Sputum samples collected were effectively treated with 2% citrate buffer (NALC-NaOH, provided by Shanghai Xuanya Biotechnology Co., Ltd., Shanghai, China) and sterile phosphate buffered saline (PBS, pH 6.8, provided by Shanghai Xinyu Biological Technology Co., Ltd., Shanghai, China), followed by centrifugation. Next, treatment liquid was added and subjected to vortex treatment. Thereafter, vortexed sputum samples (with a volume of 2 mL) were placed in a GeneXpert nucleic acid amplification instrument for fully automatic detection. About 2 h later, final test results were obtained.

#### 2.2.3. Gene Chip Technology

Sputum samples were dripped with digestive solution, vortexed, and deposited, followed by nucleic acid extraction. Instantaneous centrifugation was carried out on control by template DNA in turn, and nucleic acid amplification was conducted in a PCR amplification instrument. The resulting PCR product gradually deformed and evolved into a hybridization mixture. The mixture was preheated, hybridized, washed, and dried. Next, it was placed on a chip array for scientific scanning with a scanner, and the detection results were automatically analyzed. About 6 h was needed from nucleic acid extraction to test result obtaining.

### 2.3. Judgment Criteria

The clinical positive rate of MTB and test duration by the GeneXpert MTB/RIF, gene chip technology, and modified Roche culture method were compared. The diagnostic performance of GeneXpert MTB/RIF and gene chip technology was compared, with the modified Roche culture method as the indicator. With clinical diagnosis as the gold standard, the diagnostic performance of GeneXpert MTB/RIF, gene chip technology, and modified Roche culture method was compared, mainly including sensitivity (number of true positives/(number of true positives + number of false negatives) 100.00%), specificity (number of true negatives/(number of true negatives + number of false positives 100.00%), accuracy, positive predictive value (PPV), negative predictive value (NPV), and Kappa value. With the results of solid culture as evaluation standards, the performance of GeneXpert MTB/RIF, gene chip technology, and modified Roche culture method in detecting drug susceptibility of MTB, mainly the susceptibility to isoniazid (INH) and RIF, was analyzed.

### 2.4. Statistical Analysis

Statistical Product and Service Solutions (SPSS) 25.0 (IBM, Armonk, NY, USA) was employed for calculation of all data obtained in this study. Measurement data were expressed as ($\bar{\chi }+s$) and subjected to the *t*-test. Enumeration data were expressed as % and subjected to the *χ*^2^ test. *P* < 0.05 indicated a statistical difference.

## 3. Results

### 3.1. Clinical Positive Rate of MTB and Test Duration

In contrast with the modified Roche culture method, the GeneXpert MTB/RIF and gene chip technology displayed a higher positive rate, and the GeneXpert MTB/RIF had the highest positive rate. In addition, the GeneXpert MTB/RIF and gene chip had a shorter overall duration, with GeneXpert MTB/RIF having the shortest overall duration. The clinical positive rate and overall test duration were of statistical differences among the above three methods (*P* < 0.05) (Table 1).

### 3.2. Performance in Diagnosis of MTB

#### 3.2.1. Diagnostic Performance of GeneXpert MTB/RIF and Gene Chip Technology

Compared with the gene chip technology, the GeneXpert MTB/RIF exhibited higher sensitivity and NPV, but lower specificity, PPV, and Kappa value, with statistically significant differences (*P* < 0.05) (Table 2). 35 (35/78) cases were tested positive by the modified Roche culture method, with an accuracy rate of 44.87%. It suggests that judging the diagnostic efficacy of GeneXpert MTB/RIF and gene chip technology with the modified Roche culture method as the reference index has obvious shortcomings.

#### 3.2.2. Diagnostic Performance of Three Methods

It was found in the analysis of the diagnostic performance of the three detection methods that the GeneXpert MTB/RIF had the highest diagnostic sensitivity, ideal predictive values, and the highest similarity with clinical diagnosis in results, and the differences were statistically significant (*P* < 0.05) (Table 3).

### 3.3. Performance in DST of MTB

The susceptibility of MTB to INH and RIF was tested on 35 samples. The results showed that the GeneXpert MTB/RIF and gene chip technology performed well in DST of MTB (Table 4).

## 4. Discussion

Early detection, diagnosis, and treatment play an important role in the effective control of tuberculosis transmission, with a high proportion of active tuberculosis being smear-negative tuberculosis. It has been reported in the research of Sah et al. and Menon et al. [6, 7] that the GeneXpert MTB/RIF has a positive rate of about 28–41% in detecting smear-negative pulmonary TB samples, consistent with the results of this study. This indicates that the GeneXpert MTB/RIF has high performance in clinical detection of smear-negative TB samples. Besides, the results of this study revealed that with the modified Roche culture method as the evaluation index, the clinical performance of GeneXpert MTB/RIF and gene chip technology in detecting MTB could not be effectively analyzed. Hence, the clinical diagnosis should be taken as the evaluation index, and it was found that the GeneXpert MTB/RIF results showed significant similarity with clinical diagnosis. However, 34 false positive cases were detected by GeneXpert MTB/RIF in this study. It may be because sputum samples of patients display a low MTB burden, which is in line with the research results of Elbrolosy et al. [8]. For these reasons, the GeneXpert MTB/RIF and gene chip technology can be combined for joint diagnosis to further enhance the performance in diagnosis of MTB, which is conducive to the evaluation of false positive diagnostic results.

In the past, drug susceptibility has been qualitatively assessed usually on the basis of the culture of MTB. Despite a relatively advanced culture system, the overall culture time of MTB is long, usually about 14 d. It was discovered in this study that the test duration of GeneXpert MTB/RIF and gene chip technology for the final acquisition of drug resistance of MTB was 2 h and 6 h, respectively, showing obvious advantages, which is consistent with the research results of Hashmi et al. [9]. The reason is that the GeneXpert MTB/RIF can execute automatic detection and DST of MTB, but it cannot effectively detect nontuberculosis mycobacteria (NTM) and TB with resistance to INH, in line with the findings by Tang and Solanki et al. [10, 11]. However, such a deficiency can be effectively made up by the gene chip technology. The gene chip technology performs better in detecting TB with resistance to INH, and meanwhile, it has high diagnostic sensitivity and specificity in isoniazid-resistant (HR)-TB [12]. Relevant studies have manifested that related studies of NTM-induced diseases are obviously increasing in China and other countries. The results of this study revealed that the infection observation rate of HR-TB disease and NTM disease was relatively low. However, the gene chip technology and modified Roche culture method had ideal and consistent diagnostic performance, and the gene chip technology can be regarded as a scientific approach for diagnosing the above two diseases. This study has the following limitations: its efficacy is not well assessed in patients <18 years of age, the sample size of the study is small, this study is not a double-blind study, and (4) this study is not a multicentre study.

## 5. Conclusion

In conclusion, the final clinical diagnosis should always be regarded as the gold standard in MTB diagnosis. Compared with the modified Roche culture method, the GeneXpert MTB/RIF and gene chip technology have more ideal diagnostic performance. However, the detection by GeneXpert MTB/RIF and gene chip technology is relatively expensive. Besides, a simple molecular biological method probably leads to certain misdiagnosis or missed diagnosis of the disease. Hence, various detection methods can be combined for diagnosis, so as to improve the accuracy of clinical diagnosis.

## Figures and Tables

**Table 1:** Probability of clinical positive detection of *Mycobacterium tuberculosis* and detection time (*n* (%)).

Group	Positive result	Negative result	Positive rate (%)	Overall length of testing
Modified Roche culture method	35	85	29.17	2–6 weeks
GeneXpert MTB/RIF	48	72	40.00	2 hours
Gene chip technology	39	81	32.50	6 hours

**Table 2:** Diagnostic efficacy of GeneXpert MTB/RIF and gene chip technology (*n* (%)).

Group		Modified Roche culture method		Sensitivity (%)	Specificity (%)	PPV	NPV	Kappa value
		+	−					
GeneXpert MTB/RIF	+	28	20	77.78	76.47	57.57	88.57	0.623
	−	8	65					
Gene chip technology	+	27	12	75.00	85.71	68.57	65.71	0.643

**Table 3:** Diagnostic efficacy of three detection methods (*n* (%)).

Group		Clinical diagnosis		Sensitivity	Specificity	PPV	NPV	Kappa value
		+	−					
Modified Roche culture method	+	35	0	44.87	98.72	100.00	48.72	0.473
	−	43	42					
GeneXpert MTB/RIF	+	44	4	56.41	100.00	91.67	53.85	0.533
	−	38	34					
Gene chip technology	+	39	0	50.00	100.00	100.00	50.83	0.523

**Table 4:** Drug sensitivity test efficacy of *Mycobacterium tuberculosis* (*n* (%)).

Group		Isoniazid conventional DST			Rifampicin conventional DST	
				Sensitive cases	Resistant cases	Sensitive cases	Resistant cases
Modified Roche culture method	Sensitive cases			29	0	27	3
	Resistant cases			1	5	2	3
GeneXpert MTB/RIF	Sensitive cases			—	—	31	0
	Resistant cases			—	—	0	4
Gene chip technology	Sensitive cases			30	0	31	0
	Resistant cases			0	5	0	4

## Data Availability

The datasets used and analyzed during the current study are available from the corresponding author upon request.
